This article has been retracted.

# N6-methyladenosine reader YTH N6-methyladenosine RNA binding protein 3 or insulin like growth factor 2 mRNA binding protein 2 knockdown protects human bronchial epithelial cells from hypoxia/reoxygenation injury by inactivating p38 MAPK, AKT, ERK1/2, and NF-κB pathways

**DOI:** 10.1080/21655979.2021.1999550

**Published:** 2022-05-19

**Authors:** Kun Xiao, Pengfei Liu, Peng Yan, Yanxin Liu, Licheng Song, Yuhong Liu, Lixin Xie

**Affiliations:** a College of Pulmonary & Critical Care Medicine, Chinese People’s Liberation Army (Pla) General Hospital, Beijing, China; b Medical School of Chinese People’s Liberation Army (Pla), Beijing, China

**Keywords:** N6-methyladenosine, YTHDF3, IGF2BP2, lung, injury, hypoxia, reoxygenation

## Abstract

Lung ischemia/reperfusion (I/R) injury (LIRI) is a common complication after lung transplantation, embolism, and trauma. N6-methyladenosine (m6A) methylation modification is implicated in the pathogenesis of I/R injury. However, there are no or few reports of m6A-related regulators in LIRI till now. In this text, dysregulated genes in lung tissues of LIRI rats versus the sham group were identified by RNA sequencing (RNA-seq). RNA-seq outcomes revealed that only YTH N6-methyladenosine RNA binding protein 3 (YTHDF3) and insulin-like growth factor 2 mRNA-binding protein 2 (IGF2BP2) were differentially expressed in the LIRI versus sham group among 20 m6A-related regulators. Next, the functions and molecular mechanisms of YTHDF3 and IGF2BP2 in LIRI were investigated in a hypoxia/reoxygenation-induced BEAS-2B cell injury model *in vitro*. Results showed that YTHDF3 or IGF2BP2 knockdown attenuated hypoxia/reoxygenation-mediated inhibitory effects on cell survival and cell cycle progression and inhibited hypoxia/reoxygenation-induced cell apoptosis and pro-inflammatory cytokine secretion in BEAS-2B cells. Genes that could be directly regulated by YTHDF3 or IGF2BP2 were identified based on prior experimental data and bioinformatics analysis. Moreover, multiple potential downstream pathways of YTHDF3 and IGF2BP2 were identified by the Kyoto Encyclopedia of Genes and Genomes (KEGG) and Gene Ontology (GO) enrichment analysis of the above-mentioned genes. Among these potential pathways, we demonstrated that YTHDF3 or IGF2BP2 knockdown inhibited hypoxia/reoxygenation-activated p38, ERK1/2, AKT, and NF-κB pathways in BEAS-2B cells. In conclusion, YTHDF3 or IGF2BP2 knockdown weakened hypoxia/reoxygenation-induced human lung bronchial epithelial cell injury by inactivating p38, AKT, ERK1/2, and NF-κB pathways.

## Highlights

- YTHDF3 and IGF2BP2 were dysregulated in lung tissues of rats after LIRI.
- YTHDF3 knockdown alleviated hypoxia/reoxygenation-induced BEAS-2B cell injury.
- IGF2BP2 loss mitigated hypoxia/reoxygenation-induced BEAS-2B cell injury.
- Potential targets and downstream pathways of YTHDF3 and IGF2BP2 were identified.
- YTHDF3 and IGF2BP2 positively regulated p38, ERK1/2, AKT, and NF-κB pathways.

## Introduction

Lung ischemia/reperfusion injury (LIRI), a pathological process caused by the deficiency and subsequent reperfusion of oxygen and blood to the lung, is characterized by epithelial/endothelial dysfunction/injury and inflammatory cytokine release [1-3]. It is a common complication after lung transplantation, embolism, trauma, resuscitation after hemorrhagic shock, and cardiopulmonary bypass cardiac surgery, and can seriously threaten the health and life of patients who underwent these diseases or events [1,4,5]. However, current therapeutic strategies are limited to supportive care and cannot specifically and effectively prevent LIRI in clinical trials [1,3]. LIRI is a complex pathological situation, which involves a cascade of biochemical, molecular, and cellular events [1,2].

N6-methyladenosine (m6A) methylation, the most abundant reversible inner modification on RNA of eukaryotes, has emerged as one of the crucial players in the regulation of gene expression and various pathophysiologic processes in recent years [6]. It is reported that m6A methylation levels of RNA can be manipulated by some methyltransferases (m6A ‘writers’) and demethylases (m6A ‘erasers’), and the fate and biological functions of m6A methylated RNA can be modulated by some special RNA binding proteins (m6A ‘readers’) [6,7]. Recently, accumulating study shows that m6A regulators are involved in the regulation of ischemia/reperfusion (I/R)-induced injury in multiple organs, such as the heart, brain, and kidney [8]. For instance, the depletion of methyltransferase 14, N6-adenosine-methyltransferase subunit (METTL14) protected the kidney from I/R injury through targeting Yes-associated protein 1 [9]. The m6A eraser FTO alpha-ketoglutarate dependent dioxygenase (FTO) was low expressed and alkB homolog 5, RNA demethylase (ALKBH5) was highly expressed in the cerebral cortex of rats after cerebral I/R injury and oxygen–glucose deprivation/reoxygenation (OGD/R)-treated primary cerebral cortical neurons [10]. Moreover, ALKBH5 and FTO protected cerebral cortical neurons from OGD/R-induced cell injury [10]. However, the roles of m6A regulators in LIRI are poorly defined.

It is well known to us that lung can be perfused by pulmonary and bronchial circulation vascular systems [11]. Clamping the pulmonary hilum can lead to ischemia by stopping both pulmonary and bronchial circulation systems [11]. Moreover, capillary endothelial or alveolar/bronchial epithelial cells have been found to be injured in I/R-treated human, rabbit, and rat lung tissues [12-14]. For instance, Almeida *et al*. demonstrated that I/R treatment led to the notable increase of the apoptotic percentage of bronchial epithelial cells in the lung tissues of rats [15]. BEAS-2B, a human bronchial epithelial cell line, has been used to examine the molecular basis of LIRI *in vitro* [16-18]. For example, OGD/R exposure triggered the notable reduction of cell survival activity in BEAS-2B cells, and nuclear factor E2-related factor 2 (Nrf2) exerted a protective effect in the LIRI mouse model and OGD/R-induced BEAS-2B cell injury model [16].

In this project, high-throughput RNA sequencing (RNA-seq) technology was used to identify differentially expressed genes in lung tissues of LIRI rats versus the sham group. These dysregulated genes might be closely linked with the pathogenesis of LIRI. Given the vital roles of m6A-related regulators in tissue I/R injury, we further examined the expression patterns of 20 m6A-related regulators in lung tissues of LIRI rats versus the sham group based on RNA-seq data. Among these 20 m6A regulators, only two m6A readers (YTH N6-methyladenosine RNA binding protein 3 (YTHDF3) and insulin-like growth factor 2 mRNA-binding protein 2 (IGF2BP2)) [19,20] were identified to be differentially expressed in the LIRI group compared to the sham group, suggesting the close association of YTHDF3/IGF2BP2 and LIRI pathogenesis. Thus, the roles of IGF2BP2 and YTHDF3 in LIRI were further investigated in the hypoxia/reoxygenation-induced BEAS-2B cell injury model *in vitro*. Moreover, bioinformatics analysis suggested that YTHDF3/IGF2BP2 might participate in the regulation of MAPK, PI3K-AKT, TNF, AKT, ERK1/ERK2, and NF-κB pathways. p38 MAPK pathway, one of the most frequently studied MAPK pathways, has been reported to be implicated in LIRI responses [21,22]. Also, AKT, ERK1/ERK2, and NF-κB pathways play crucial roles in LIRI [23-25]. Thus, we further explored whether IGF2BP2 or YTHDF3 could exert its functions by regulating p38 MAPK, AKT, ERK1/ERK2, and NF-κB pathways in the hypoxia/reoxygenation-induced BEAS-2B cell injury model *in vitro*.

## Materials and methods

### Animal experiments

The animal experiments were performed with the approval of the Animal Care and Use Committee of the People’s Liberation Army General Hospital. A LIRI model was established as previously described [26]. Sprague–Dawley (SD) rats (n = 6, male, 7–8 weeks old, 220–280 g) were purchased from Beijing HFK Bioscience Co., Ltd. (Beijing, China) and left to acclimatize to the experimental environment for 1 week. Rats were randomly divided into sham and LIRI groups with 3 rats per group. After being anesthetized with urethane (*i.p*.), SD rats were endotracheally intubated and ventilated using an animal ventilator under the conditions: respiratory rate of 70 breaths/min, tidal volume of 20 ml/kg, and inspiratory/expiratory ratio of 1:1. After thoracotomy, the left pulmonary hilum of rats in the LIRI group was clamped for 60 min using the noninvasive vascular clips, followed by the 120 min of reperfusion treatment. Rats in the sham group only received the thoracotomy without hilar occlusion. Finally, rats were euthanized and left lung tissues were isolated for following reverse transcription-quantitative PCR (RT-qPCR) assay and RNA sequencing (RNA-seq) analysis. The detailed information of animal experiments will be reported elsewhere (manuscript in preparation). RNA-seq was performed on the Illumina PE150. FPKM (fragments per kilobases per million fragments) method was used to normalize the counts of sequencing reads. Genes were defined to be differentially expressed at the |log_2_FoldChange| > 1 and adjusted *P* (padj) value < 0.05. Gene Ontology (GO) and Kyoto Encyclopedia of Genes and Genomes (KEGG) pathway enrichment analysis was performed using the online website (http://kobas.cbi.pku.edu.cn/kobas3).

### Cell culture

BEAS-2B cells were purchased from American Type Culture Collection (ATCC, Manassas, VA, USA) and cultured in DMEM/F-12 medium (Thermo Fisher Scientific, Waltham, MA, USA) supplemented with 10% fetal bovine serum (Thermo Fisher Scientific), 2 mM L-glutamine (Thermo Fisher Scientific), 100 U/mL penicillin (Thermo Fisher Scientific), and 100 mg/mL streptomycin (Thermo Fisher Scientific).

### Reagents and cell transfection

Three small interference RNAs (siRNAs) targeting YTHDF3 (si-YTHDF3#1, si-YTHDF3#2, si-YTHDF3#3) or IGF2BP2 (si-IGF2BP2#1, si-IGF2BP2#2, si-IGF2BP2#3) and a scrambled siRNA control (si-NC) were purchased from GenePharma Co., Ltd. (Shanghai, China). These siRNAs were transfected into BEAS-2B cells using Lipofectamine 3000 reagent (Thermo Fisher Scientific). The sequences of these siRNAs were presented in Table 1.

**Table 1.** The sequences of primers and oligonucleotides

Gene name	Primer sequence (5ʹ-3ʹ)
YTHDF3 (Rat)	F: TCAACCAGAACAATGGAACAGG
	R: GAACGGTAAGCTGCATCCAAA
IGF2BP2 (Rat)	F: CCCCCTATCACCCATTTGCT
	R: TCGAGCCAGCTGTTTGATGT
β-actin (Rat)	F: TCAGGTCATCACTATCGGCAAT R: CACCCGCGAGTACAACCTTC
	R: AAAGAAAGGGTGTAAAACGCA
YTHDF3 (Human)	F: TCAGAGTAACAGCTATCCACCA
	R: GGTTGTCAGATATGGCATAGGCT
IGF2BP2 (Human)	F: AGCCTGTCACCATCCATGC
	R: CTTCGGCTAGTTTGGTCTCATC
β-actin (Human)	F: CTCCATCCTGGCCTCGCTGT
	R: GCTGTCACCTTCACCGTTCC
	Oligonucleotide (Sense sequence)
si-YTHDF3#1	GGUGGAUUUCACCAGUUAAUG
si-YTHDF3#2	AGAUGGUGUAUUUAGUCAACC
si-YTHDF3#3	GGGCAAAUUUGAAGUUAAAUG
si-IGF2BP2#1	GCCGUUGUCAACGUCACAUAU
si-IGF2BP2#2	AGCGCAAGAUCAGGGAAAUUG
si-IGF2BP2#3	AGAUAGAGAUUAUGAAGAAGC

### Reverse transcription -quantitative polymerase chain reaction (RT-qPCR)

RT-qPCR was carried out as previously described [27,28]. Briefly, total RNA was extracted from lung tissues and BEAS-2B cells using Trizol reagent (Thermo Fisher Scientific) following the manufacturer’s protocols. Next, cDNA first strand was synthesized using RevertAid First-Strand cDNA Synthesis Kit (Thermo Fisher Scientific) and quantitative PCR reaction was performed using SYBR Select Master Mix (Thermo Fisher Scientific) referring to the instructions of manufacturer on ABI QuantStudio 6 Felx Real-Time System (Thermo Fisher Scientific). The primers were obtained from Sangon Biotech Co., Ltd. (Shanghai, China). The primer sequences were shown in Table 1. β-actin was used as a housekeeping gene. The relative expression levels of genes were measured using the 2^−ΔΔCt^ method.

### Cell counting kit-8 assay

The viability of BEAS-2B cells was assessed by CCK-8 assay using the Cell Counting Kit-8 (CCK-8) assay kit (MedChemExpress, Monmouth Junction, NJ, USA) following the manufacturer’s instructions as previously described [29,30]. Briefly, transfected or non-transfected cells were inoculated into 96-well plates. At the indicated time points after treatment, 10 μl of CCK-8 solution was added to each well of the plates and incubated for an additional 3 h. Next, the absorbance was examined at 450 nm. Cell viability = (OD _experiment group –_ OD _blank group_)/(OD_normoxia group_ (0 h) – OD _blank group_ (0 h)) *100%.

### Cell apoptotic rate detection

The apoptotic rate of BEAS-2B cells was determined using an Annexin V-FITC Apoptosis Detection Kit (Beyotime Biotechnology, Shanghai, China) according to the manufacturer’s protocols as described previously [31,32]. Briefly, cells resuspended in Annexin V-FITC binding solution (195 μL) were co-incubated with Annexin V-FITC solution (5 μL) and Propidium Iodide (PI) solution (10 μL) for 15 min at room temperature under dark conditions. Finally, cell apoptotic rate (Q1-UR+Q1-LR) was examined using flow cytometry (BD Biosciences, San Jose, CA, USA).

### Cell cycle distribution pattern detection

Cell cycle distribution pattern was determined referring to the method as previously described [33,34]. Briefly, BEAS-2B cells were fixed overnight with pre-cold 70% ethanol at 4°C. After washed, cells were co-incubated with the solution containing RNase A (100 µg/ml), PI (50 µg/ml), and 0.1% Triton X-100 for 0.5 h at room temperature under dark conditions. Next, the cell cycle distribution pattern was examined via flow cytometry (BD Biosciences).

### ELISA assay

Tumor necrosis factor-alpha (TNF-α) and interleukin 1 beta (IL-1β) secretion levels in BEAS-2B cell supernatants were determined using corresponding ELISA kits (Elabscience Biotechnology Co., Ltd., Wuhan, China) according to the manufacturer’s protocols as previously described [35,36].

### Western blot analysis

Western blot analysis was carried out as previously reported [37,38]. Briefly, protein was extracted from BEAS-2B cells using the RIPA lysis buffer (Beyotime Biotechnology) supplemented with phenylmethanesulfonyl fluoride (PMSF, Aladdin, Shanghai, China) and sodium orthovanadate (phosphatase inhibitor, Beyotime Biotechnology), and then quantified using the Enhanced BCA Protein Assay Kit (Beyotime Biotechnology). Equal amounts of protein extracts were separated through 12% sodium dodecyl sulfate-polyacrylamide gel electrophoresis and transferred to polyvinylidene fluoride membranes (Millipore, Bedford, MA, USA). Next, nonspecific protein signals on the membranes were blocked with 1% BSA (for phosphorylated proteins) or 5% nonfat milk (for non-phosphorylated proteins) for 2 h at room temperature. Next, the membranes were incubated overnight at 4°C with primary antibodies against AKT (1:500 dilution; ab8805), p-AKT (1:600 dilution; ab38449), ERK1/2 (1:10,000 dilution; ab184699), p-ERK1/2 (1:1000 dilution; ab201015), p38 (1:2000 dilution; ab170099), p-p38 (1:1000 dilution; ab178867), p65 (1:20,000 dilution; ab32536), p-p65 (1:1000 dilution; ab76302) and β-actin (1:2000 dilution; ab8227). All the primary antibodies were purchased from Abcam Inc. (Cambridge, UK). Next, the membranes were probed with horseradish peroxidase-conjugated goat anti-rabbit secondary antibody (1:5000 dilution; BA1054; Boster Biological Technology, Wuhan, China) for 1 h at room temperature. Finally, protein bands were developed using the Super ECL Plus Western Blotting Substrate (Applygen Technologies, Beijing, China).

### Statistical analysis

Data were analyzed using GraphPad Prism 7 software (GraphPad Software, Inc., San Diego, CA, USA) and expressed as mean ± standard deviation. Difference comparisons between groups were performed using Student’s *t-*test. Difference analysis among groups was conducted by one-way Analysis of Variance (ANOVA, Dunnet post-hoc test) or two-way ANOVA (Tukey post hoc test). The difference was considered statistically significant at the *P* value less than 0.05.

## Results

In this text, the transcriptomic difference in lung tissues of LIRI rats versus the sham group was identified by RNA-seq technology to have an in-depth insight into the molecular basis of LIRI. M6A modification and m6A-related regulators have been found to be closely linked with the pathogenesis of I/R injury. To identify m6A-related regulators that might play vital roles in LIRI, the expression patterns of 20 m6A-related regulators were examined based on RNA-seq analysis. Among the 20 m6A-related regulators, only YTHDF3 and IGF2BP2 were found to be differentially expressed in lung tissues of LIRI rats versus the sham group, suggesting that YTHDF3 and IGF2BP2 might play vital roles in the development of LIRI. It has been reported that lung I/R treatment can lead to the injury of lung bronchial epithelial cells. Hence, a hypoxia/reoxygenation-induced BEAS-2B cell injury model was established to explore the roles and downstream regulatory mechanisms of YTHDF3 and IGF2BP2 in LIRI *in vitro*. In our project, the influences of YTHDF3 or IGF2BP2 knockdown on hypoxia/reoxygenation-induced BEAS-2B cell injury were assessed by cell viability, cell cycle progression, cell apoptosis, and pro-inflammatory cytokine secretion patterns. Next, genes that could be directly regulated by YTHDF3 or IGF2BP2 were identified based on bioinformatics prediction analysis and previous experimental data. Moreover, KEGG and GO enrichment analysis of the above-mentioned possible targets of YTHDF3 or IGF2BP2 was performed to identify the potential downstream signaling pathways of YTHDF3 or IGF2BP2. Among the pathways that could be significantly enriched by the above-mentioned potential targets of YTHDF3 or IGF2BP2, we further explored the effects of YTHDF3 or IGF2BP2 knockdown on AKT, NF-κB, ERK1/2, and P38 pathways in the hypoxia/reoxygenation-induced BEAS-2B cell injury model because these 4 pathways have been found to be implicated in the development of LIRI.

### Identification and GO/KEGG enrichment analysis of differentially expressed genes in lung tissues of LIRI rats versus the sham group

To screen out the vital genes implicated in the pathogenesis of LIRI, comparative transcriptome analysis was performed by RNA-seq in lung tissues of LIRI and sham rats. The detailed experimental outcomes of animal experiments will be presented elsewhere (manuscript in preparation). RNA-seq outcomes showed that plenty of genes were differentially expressed in the LIRI group versus the sham group (Figure 1a, Supplementary Table 1). GO enrichment analysis revealed that these differentially expressed genes were involved in the regulation of a host of biological processes including transcription, cell morphogenesis, cell population proliferation, phosphatidylinositol-mediated signaling, mitochondrial membrane potential, ERK1/ERK2, and JNK cascade, protein tyrosine kinase activity, cellular response to interleukin-1/tumor necrosis factor/hypoxia, I-kappaB kinase/NF-kappaB (NF-κB) signaling, cell growth, cell cycle progression, cytokinesis and apoptotic signaling pathway (Supplementary Table 2 sheet 1 and Figure 1b). KEGG enrichment outcomes showed that these differentially expressed genes were significantly enriched in multiple pathways such as bacterial invasion of epithelial cells, MAPK/HIF-1 signaling pathway, phosphatidylinositol signaling system, carbohydrate digestion and absorption, cellular senescence, and inflammatory mediator regulation of TRP channels (Supplementary Table 2 sheet 2 and Figure 1c). Considering the close association of m6A methylation modification and the etiology of I/R injury, we further explored whether 20 m6A-related regulators (methyltransferase 3, N6-adenosine-methyltransferase complex catalytic subunit (METTL3), methyltransferase 14, N6-adenosine-methyltransferase subunit (METTL14), methyltransferase 16, N6-methyladenosine (METTL16), WT1 associated protein (WTAP), vir like m6A methyltransferase associated (KIAA1429), RNA binding motif protein 15 (RBM15), RNA binding motif protein 15B (RBM15B), FTO, ALKBH5, YTH N6-methyladenosine RNA binding protein 1 (YTHDF1), YTH N6-methyladenosine RNA binding protein 2 (YTHDF2), YTH N6-methyladenosine RNA binding protein 3 (YTHDF3), YTH domain containing 1 (YTHDC1), YTH domain containing 2 (YTHDC2), heterogeneous nuclear ribonucleoprotein A2/B1 (HNRNPA2B1), heterogeneous nuclear ribonucleoprotein C (HNRNPC), FMRP translational regulator 1 (FMR1), eukaryotic translation initiation factor 3 subunit A (eIF3), IGF2BP2, insulin-like growth factor 2 mRNA binding protein 3 (IGF2BP3) were differentially expressed in the LIRI group versus the sham group. Among these m6A regulators, only YTHDF3 (12.18-fold up-regulation) and IGF2BP2 (15.14-fold down-regulation) were identified to be differentially expressed in the LIRI group versus the sham group. Following RT-qPCR assay also verified the differential expression of YTHDF3 and IGF2BP2 in the LIRI group compared with the sham group (Figures 1d and 1e).

**Figure 1.** **Identification of differentially expressed genes in lung tissues of LIRI rats versus the sham group**. (a) Volcano plots of differentially expressed genes in the LIRI versus sham group. (b) Partial GO enrichment outcomes of differentially expressed genes in the LIRI versus sham group. (c) Partial KEGG enrichment outcomes of differentially expressed genes in the LIRI versus sham group. (d and e) The expression levels of YTHDF3 and IGF2BP2 were determined by RT-qPCR assay.

### Establishment of an in vitro hypoxia/reoxygenation injury model in BEAS-2B cells

CCK-8 assay revealed that the viability of BEAS-2B cells was time-dependently reduced in response to hypoxia/reoxygenation treatment (Figure 2a). Moreover, hypoxia/reoxygenation treatment triggered a time-dependent elevation of cell apoptotic rate in BEAS-2B cells (Figure 2b). Additionally, hypoxia/reoxygenation exposure time-dependently facilitated IL-1β and TNF-α secretion in BEAS-2B cells (Figures 2c and 2d). These data suggested that hypoxia/reoxygenation exposure could cause BEAS-2B cell injury. Given the moderate injury and highest IL-1β and TNF-α secretion after 6 h/6 h of hypoxia/reoxygenation treatment, this condition was used to establish the *in vitro* hypoxia/reoxygenation injury model in BEAS-2B cells.

**Figure 2.** **Establishment of an *in vitro* hypoxia/reoxygenation injury model in BEAS-2B cells**. (a-d) BEAS-2B cells were exposed to hypoxic conditions for 0, 2, 4, 6, or 12 h, and then maintained in normoxic conditions (reoxygenation) for the same treatment time-period with hypoxia. (a) Cell viability was measured by CCK-8 assay. (b) Cell apoptotic rate was measured using flow cytometry. (c and d) The secretion levels of IL-1β and TNF-α were examined by ELISA assay.

### YTHDF3 or IGF2BP2 knockdown improved cell viability, facilitated cell cycle progression, hindered cell apoptosis, and inhibited IL-1β and TNF-α secretion in BEAS-2B cells exposed to hypoxia/reoxygenation

Next, 3 siRNAs targeting YTHDF3 (si-YTHDF3#1, si-YTHDF3#2, and si-YTHDF3#3) or IGF2BP2 (si-IGF2BP2#1, si-IGF2BP2#2, and si-IGF2BP2#3) were synthesized to investigate the functions of YTHDF3 and IGF2BP2. Results showed that the transfection of si-YTHDF3#1, si-YTHDF3#2, or si-YTHDF3#3 led to the notable reduction of YTHDF3 level in BEAS-2B cells (Supplementary Fig. 1A). Hence, an equal proportion mixture of si-YTHDF3#1, si-YTHDF3#2, and si-YTHDF3#3, named si-YTHDF3, was used in the subsequent experiments. Also, there was a marked decrease of IGF2BP2 level in BEAS-2B cells transfected with si-IGF2BP2#1, si-IGF2BP2#2, or si-IGF2BP2#3 than in si-NC-transfected cells (Supplementary Fig. 1B). Thus, the 1:1:1 mixture of si-IGF2BP2#1, si-IGF2BP2#2, and si-IGF2BP2#3, named si-IGF2BP2, was used in the following experiments.

CCK-8 assay showed that YTHDF3 or IGF2BP2 loss markedly enhanced cell viability in BEAS-2B cells after hypoxia/reoxygenation exposure (Figure 3a). Moreover, YTHDF3 or IGF2BP2 knockdown led to the conspicuous reduction of cell percentage in the G1 phase and noticeable increase of cell proportion in S and G2 phases in BEAS-2B cells after hypoxia/reoxygenation treatment, suggesting that YTHDF3 or IGF2BP2 depletion promoted cell cycle progression in hypoxia/reoxygenation-exposed BEAS-2B cells (Figure 3b). Additionally, YTHDF3 knockdown triggered an approximately 0.43-fold reduction in cell apoptotic rate in BEAS-2B cells exposed to hypoxia and reoxygenation (Figure 3b). Also, there was an about 0.26-fold decrease of cellular apoptotic percentage in BEAS-2B cells treated with hypoxia and reoxygenation following the depletion of IGF2BP2 (Figure 3b). Lung I/R can induce excessive pulmonary inflammation and cause lung tissue damage via the production of pro-inflammatory cytokines [39]. TNF-α and IL-1β are two frequently studied pro-inflammatory cytokines in acute injury models including LIRI [40,41]. Previous studies showed that the deficiency or inhibition of TNF-α and IL-1β could notably alleviate LIRI [40,42,43]. Moreover, An *et al*. demonstrated that the intravenous injection of anti-TNF-α antibody inhibited the apoptosis of lung epithelial cells in rats after I/R of the small intestine [14]. Thus, the effects of YTHDF3 or IGF2BP2 knockdown on IL-1β and TNF-α secretion were examined through ELISA assay. Results showed that YTHDF3 or IGF2BP2 loss noticeably inhibited IL-1β and TNF-α secretion in hypoxia/reoxygenation-treated BEAS-2B cells (Figures 3c and 3d). These data suggested that YTHDF3 or IGF2BP2 knockdown protected BEAS-2B cells against hypoxia/reoxygenation-induced cell damage.

**Figure 3.** **YTHDF3 or IGF2BP2 knockdown improved cell viability, facilitated cell cycle progression, hindered cell apoptosis, and inhibited IL-1β and TNF-α secretion in BEAS-2B cells treated with hypoxia/reoxygenation**. (a) BEAS-2B cells in the H/R groups were transfected with or without si-NC, si-YTHDF3, or si-IGF2BP2 and then exposed to hypoxic conditions for 6 h and normoxic conditions for the remaining time. Cells prior to hypoxic treatment were named as the 0-h groups. Cell viability was examined by CCK-8 assay. (b-d) BEAS-2B cells were transfected with or without si-NC, si-YTHDF3, or si-IGF2BP2 for 48 h and then treated with normoxia or hypoxia/reoxygenation. Hypoxia//reoxygenation conditions: 6 h of exposure to hypoxic conditions (5% CO_2_, 94%N_2_, 1% O_2_) and another 6 h of normoxic (95% air, 5% CO_2_) treatment. (b) Cell apoptotic rate and cell cycle distribution patterns were measured using flow cytometry. (c and d) IL-1β and TNF-α secretion levels were determined by ELISA assay.

### Identification of YTHDF3 and IGF2BP2 downstream regulatory pathways

Bioinformatics prediction analysis (http://m6a2target.canceromics.org/#/) revealed that 1201 protein-coding genes could directly bind with YTHDF3 (Supplementary Table 3 sheet 1). Moreover, a recent study showed that YTHDF3 knockdown could trigger the differential expression of 1174 protein-coding genes in colorectal cancer cells [44] (Supplementary Table 3 sheet 2). Combined with the m6a2target prediction data and the previous experimental outcomes, 87 common genes were identified by Venn analysis (Supplementary Table 3 sheet 3, Figure 4a). These genes had a high possibility to be directly regulated by YTHDF3. KEGG enrichment analysis showed that MAPK, PI3K-AKT, and TNF signaling pathways could be markedly enriched by these 87 common genes (Supplementary Table 4 sheet 1, Figure 4b). GO_biological process enrichment analysis suggested that these 87 potential YTHDF3 targets mainly participated in the regulation of apoptotic progress, AKT signaling, ERK1/ERK2 cascades, and cell proliferation (Supplementary Table 4 sheet 2, Figure 4c). The top 30 KEGG pathways and biological processes enriched by these 87 potential YTHDF3 targets were presented in Figure 4b and Figure 4c, respectively. Moreover, the prediction analysis by the Starbase database (http://starbase.sysu.edu.cn/rbpClipRNA.php?source=mRNA&flag=RBP&clade=mammal&genome=human&assembly=hg19&RBP=IGF2BP2&clipNum=&panNum=&target=) revealed that IGF2BP2 could directly bind with 15,705 protein-coding genes (Supplementary Table 5). Additionally, the differential expression analysis of the GSE146726 dataset showed that IGF2BP2 loss led to the differential expression of 1040 or 920 genes in UMUC3 or J82 bladder cancer cells, respectively (Supplementary Table 6). Next, 206 common genes were identified by Venn analysis of genes in Supplementary Table 5 and Table 6 (Figure 4d). These 206 genes might be the direct targets of IGF2BP2. KEGG enrichment analysis showed that these 206 potential IGF2BP2 targets were significantly enriched in multiple KEGG pathways including apoptosis, MAPK, TNF, and PI3K-AKT signaling pathways (Supplementary Table 7 sheet 1, Figure 4e), suggesting that IGF2BP2 might be involved in the regulation of these pathways. GO enrichment analysis revealed that these 206 genes functioned as crucial players in various biological processes such as cellular response to hypoxia, cell proliferation, cell apoptosis, and regulation of MAPK cascade, NF-kappaB (NF-κB) signaling, and JNK cascade (Supplementary Table 7 sheet 2, figure 4f). The top 30 KEGG pathways and biological processes enriched by the 206 potential IGF2BP2 targets were presented in Figures 4e and 4f, respectively.

**Figure 4.** **Identification of YTHDF3 and IGF2BP2 downstream regulatory pathways**. (a) Identification of potential YTHDF3 targets. Sheet 1: m6a2target (http://m6a2target.canceromics.org/#/)-predicted protein-coding genes that could directly bind with YTHDF3. Sheet 2: Differentially expressed protein-coding genes after YTHDF3 knockdown in colorectal cancer cells. (b) The top 30 KEGG pathways enriched by the 87 potential YTHDF3 targets. (c) The top 30 biological processes enriched by the 87 potential YTHDF3 targets. (d) Identification of potential IGF2BP2 targets. List 1: Potential protein-coding genes with the probability to directly bind with IGF2BP2 were predicted by the Starbase database. List 2: Differentially expressed genes in IGF2BP2-depleted UMUC3 cells compared to the control group. List 3: Differentially expressed genes in IGF2BP2-depleted J82 cells versus the control group. (e) The top 30 KEGG pathways enriched by the 206 potential IGF2BP2 targets. (f) The top 30 biological processes enriched by the 206 possible IGF2BP2 targets.

### YTHDF3 or IGF2BP2 knockdown inhibited AKT, NF-κB, ERK1/2, and p38 pathways in hypoxia/reoxygenation-treated BEAS-2B cells

As described above, GO and KEGG enrichment analyses showed that the potential targets of YTHDF3 or IGF2BP2 might participate in the regulation of MAPK, PI3K-AKT, TNF, AKT, ERK1/ERK2, and NF-κB pathways. These pathways have been identified as vital players in a host of biological processes such as cell proliferation, differentiation, apoptosis, and motility [45-47]. p38 MAPK pathway also plays vital roles in LIRI responses [21,47,48]. Thus, the effects of YTHDF3 or IGF2BP2 knockdown on AKT, NF-κB, ERK1/2, and p38 pathways were examined in the hypoxia/reoxygenation-induced BEAS-2B cell injury model. Results showed that p-AKT, p-p65, p-ERK1/2, and p-p38 protein levels were markedly increased in BEAS-2B cells after hypoxia and reoxygenation exposure (Figure 5), suggesting that hypoxia and reoxygenation treatment could induce the activation of AKT, NF-κB, ERK1/2, and p38 pathways. Moreover, YTHDF3 or IGF2BP2 knockdown led to the notable reduction of p-AKT, p-p65, p-ERK1/2, and p-p38 protein levels in BEAS-2B cells with hypoxia and reoxygenation treatment (Figure 5), indicating that YTHDF3 or IGF2BP2 loss inhibited the AKT, NF-κB, ERK1/2, and p38 pathways in hypoxia/reoxygenation-treated BEAS-2B cells.

**Figure 5.** **YTHDF3 or IGF2BP2 knockdown inhibited the hypoxia/reoxygenation-induced activation of AKT, NF-κB, ERK1/2, and P38 pathways in BEAS-2B cells**. BEAS-2B cells were transfected with or without si-NC, si-YTHDF3, or si-IGF2BP2 for 48 h. Transfected or non-transfected cells received the treatment of normoxia or hypoxia/reoxygenation. Hypoxia/reoxygenation conditions: 6 h of exposure to hypoxic conditions (5% CO_2_, 94%N_2_, 1% O_2_) and another 6 h of normoxic (95% air, 5% CO_2_) treatment. Protein levels of AKT, p-AKT, p65, p-p65, ERK1/2, p-ERK1/2, p38, and p-p38 were measured by western blot assay.

## Discussion

YTHDF3 is a member of the YTH (YT521-B homology) domain-containing protein family (YTHDF), which also contains YTHDF1, YTHDF2, YTHDC1, and YTHDC2 [49]. Recently, YTHDC1 and YTHDF1 (two membranes of the YTHDF family) have been demonstrated to be involved in the regulation of cerebral ischemic-reperfusion injury [50,51]. YTHDF3 has been found to be co-localized exclusively with the stress granules and to be a crucial player in oxidative stress response [52,53]. Considering the close association of oxidative stress and LIRI development [3,54], we further investigated whether YTHDF3 could regulate LIRI development. Our data revealed that YTHDF3 expression was markedly up-regulated in lung tissues of LIRI rats compared to the sham group. YTHDF3 knockdown weakened the detrimental effect of hypoxia/reoxygenation on cell viability and cell cycle progression and inhibited the increase of cell apoptotic rate and pro-inflammatory cytokine (IL-1β and TNF-α) secretion levels induced by hypoxia/reoxygenation in BEAS-2B cells, suggesting that YTHDF3 loss could mitigate hypoxia/reoxygenation-induced lung epithelial cell injury.

IGF2BP2 is a vital payer in multiple biological processes such as cell proliferation, epithelial-mesenchymal transition, and metabolism [55,56]. Moreover, Zhu *et al*. pointed out that IGF2BP2 was implicated in hypoxic/ischemic brain injury [57]. Given the correlation of IGF2BP2 and hypoxic injury, we supposed that IGF2BP2 might play a vital role in LIRI. Our outcomes presented that IGF2BP2 expression was markedly reduced in lung tissues of LIRI rats versus the sham group. Moreover, IGF2BP2 depletion increased cell viability, facilitated cell cycle progression, curbed cell apoptosis, and reduced pro-inflammatory cytokine (IL-1β and TNF-α) secretion in BEAS-2B cells exposed to hypoxia/reoxygenation, indicating the protective effect of IGF2BP2 loss on hypoxia/reoxygenation-induced lung epithelial cell injury. We noticed that the alteration trends of YTHDF3 and IGF2BP2 were converse in the LIRI versus sham groups. However, the functions of YTHDF3 and IGF2BP2 were similar in hypoxia/reoxygenation-treated BEAS-2B cells. It is well known to us that gene expression levels are regulated by upstream regulatory factors and genes exert their functions by controlling downstream factors. Hence, it is reasonable that the expression alterations of YTHDF3 and IGF2BP2 were converse and the functions of YTHDF3 and IGF2BP2 were similar in our project.

As mentioned above, bioinformatics analyses suggested that YTHDF3 and IGF2BP2 might exert their functions by regulating MAPK, ERK, AKT, and NF-κB pathways. Moreover, previous studies showed that TNF-α and IL-1β could induce the activation of multiple signaling pathways, such as JNK, p38 MAPK, and NF-κB and regulate multiple biological processes, such as cell proliferation, apoptosis, and inflammatory responses [58,59]. The abnormal activation of p38 MAPK [21,60], ERK1/2 [24,61], AKT [23,62], and NF-κB [63,64] pathways have been found to be implicated in the pathogenesis of I/R injury in multiple organs including lung. For instance, the inhibition of the p38 MAPK pathway by its inhibitor FR167653 or SB239063 could alleviate LIRI [43,65,66]. The introduction of an ERK1/2 pathway inhibitor U0126 mitigated Spred2 deficiency-induced LIRI [24]. Methane weakened LIRI by reducing oxidative stress, inhibiting pro-inflammatory cytokine (*e.g*. TNF-α and IL-1β) secretion, and inactivating p38 MAPK/NF-κB/AKT signaling pathways [67]. Thus, we further investigated the effects of YTHDF3 or IGF2BP2 knockdown on these pathways in lung epithelial cells exposed to hypoxia/reoxygenation. Results showed that YTHDF3 or IGF2BP2 knockdown inhibited the activation of p38 MAPK, ERK1/2, AKT, and NF-κB pathways induced by hypoxia/reoxygenation in lung epithelial cells.

### Conclusion

Taken together, our data showed that YTHDF3 or IGF2BP2 knockdown alleviated hypoxia/reoxygenation-induced lung epithelial cell injury by inactivating p38 MAPK, ERK1/2, AKT, and NF-κB pathways, suggesting the critical roles of YTHDF3 and IGF2BP2 (two m6A readers) in the development of LIRI. It is the first study to explore the functions and molecular mechanisms of YTHDF3 and IGF2BP2 in LIRI. Moreover, a multitude of signaling pathways and targets that might be regulated by YTHDF3 or IGF2BP2 were identified. However, due to the limitation of time and funds, the effects of YTHDF3 or IGF2BP2 on LIRI progression were not investigated *in vivo*.

## Supplementary Material

Supplemental Material

## Data Availability

The data and material presented in this manuscript is available from the corresponding author on reasonable request.
